RETRACTED

# miR-126 Functions as a Tumor Suppressor in Osteosarcoma by Targeting Sox2

**DOI:** 10.3390/ijms15010423

**Published:** 2013-12-31

**Authors:** Chenglin Yang, Chunying Hou, Hepeng Zhang, Dewei Wang, Yan Ma, Yunqi Zhang, Xiaoyan Xu, Zhenggang Bi, Shuo Geng

**Affiliations:** Department of Orthopedic Surgery, the First Affiliated Hospital of Harbin Medical University, Harbin 150001, Heilongjiang, China; E-Mails: yangchenglindoctor@gmail.com (C.Y.); chunying_hou@126.com (C.H.); zhanghepengdoctor@gmail.com (H.Z.); wdw19761224@gmail.com (D.W.); mayandoctor@gmail.com (Y.M.); zhangyunqidoctor@gmail.com (Y.Z.); xxydoctor@gmail.com (X.X.); bizhenggang@163.com (Z.B.)

**Keywords:** osteosarcoma, miR-126, tumor suppressor, sex-determining region Y-box 2

## Abstract

Osteosarcoma (OS) is the most common malignant bone tumor in children and young adults, the early symptoms and signs of which are non-specific. The discovery of microRNAs (miRNAs) provides a new avenue for the early diagnosis and treatment of OS. miR-126 has been reported to be highly expressed in vascularized tissues, and is recently widely studied in cancers. Herein, we explored the expression and significance of miR-126 in OS. Using TaqMan RT-PCR analysis, we analyzed the expression of miR-126 in 32 paired OS tumor tissues and 4 OS cell lines and found that miR-126 was consistently under-expressed in OS tissues and cell lines compared with normal bone tissues and normal osteoblast cells (NHOst), respectively. As miR-126 is significantly decreased in OS tissues and cell lines, we sought to compensate for its loss through exogenous transfection into MG-63 cells with a miR-126 mimic. Ectopic expression of miR-126 inhibited cell proliferation, migration and invasion, and induced apoptosis of MG-63 cells. Moreover, bioinformatic prediction suggested that the sex-determining region Y-box 2 (Sox2) is a target gene of miR-126. Using mRNA and protein expression analysis, luciferase assays and rescue assays, we demonstrate that restored expression of Sox2 dampened miR-126-mediated suppression of tumor progression, which suggests the important role of miR-126/Sox2 interaction in tumor progression. Taken together, our data indicate that miR-126 functions as a tumor suppressor in OS, which exerts its activity by suppressing the expression of Sox2.

## 1. Introduction

Osteosarcoma (osteogenic sarcoma, OS) is the most common malignant bone tumor in children and young adults. Combined with Ewing’s sarcoma, OS represents 6% of all childhood cancers [1]. The early symptoms and signs including pain and a palpable mass are totally non-specific, leading to a delay in early diagnosis. A previous study reported that the average diagnostic delay for OS is 9 weeks, and the most common misdiagnosis is tendonitis [2]. During the past decades, although great efforts have been exerted to interpret the underlying mechanisms in OS carcinogenesis, the survival of OS reached a plateau, and the prognosis of advanced OS remains poor [3]. As the benefits from traditional chemotherapy have seemingly been maximized, novel diagnostic biomarkers and therapeutic alternatives for OS patients are needed.

RETRACTED

MicroRNAs (miRNAs) represent a new group of endogenous, small, non-coding RNAs that can modulate protein expression by regulating translational efficiency or cleavage of targets [4]. Considered to be newly important components of gene regulators, miRNAs play a critical role in the regulation networks of gene expression and are emerging as novel biomarkers of diseases [5,6]. Through completely or partially complementary with the 3′-untranslated region (3′UTR) of specific messenger RNAs, miRNAs induce various target genes, silencing and participating in various cell biological processes. Recently, numerous studies reported the association between dysregulation of miRNAs and OS, switching from profiling studies to biological demonstrations of the causal role of these small molecules in OS pathogenesis, and the possible implications as biomarkers or therapeutic tools [7]. For instance, the expression of miR-214 is constitutively up-regulated in OS tissues relative to normal bone tissues, and the higher expression of miR-214 always suggests the larger tumor size, positive metastasis, poor-response to chemistry, and shorter overall survival [8]; miR-24 could inhibit OS cell proliferation *in vitro*, and suppressed tumor growth *in vivo* [9]. Therefore, better knowledge of miRNA-mediated effects during OS carcinogenesis may provide new avenues for OS diagnostic and treatment regiments.

Recently, Namløs *et al*. compared the miRNAs expression profiles between EuroBoNeT human OS cell lines and clinical samples; they found that miR-1, miR-9, miR-18a, miR-18b, miR-126, miR-133b, miR-144, miR-195 and miR-451 were consistently decreased in both cell lines and clinical samples compared with normal bone tissues [10]. Among these miRNAs, miR-126, which is under-expressed in both cell lines and clinical samples, attracted our attention. miR-126 (also referred as miR-126-3p) is a highly conserved gene among different species [11]. As encoded by intron 7 of the epidermal growth factor-like domain 7 gene (*egfl*7), miR-126 has been reported to be highly expressed in vascularized tissues such as heart, liver, and lung, and mediates vascular functions, as well as maintaining vascular integrity [12]. More recently, the role of miR-126 in tumor progression has been widely identified. Loss of miR-126 may result in elevated tumor proliferation, migration and survival, as well as increased leukocyte adhesion and disorganized tumor vasculature [13–15]. However, the functions of miR-126 on OS cells and relative mechanisms are largely unknown.

RETRACTED

Sex-determining region Y-related high-mobility group box gene family (*Sox*) proteins are a class of transcriptional factors containing a high-mobility-group (*HMG*) domain with 50% or higher amino acid similarity to the *HMG* domain of mammalian testis determining factor *Sry* [16]. Relying on the *HMG* domain, *Sox* proteins could bind DNA in a sequence-specific manner, which causes the DNA to bend through a dramatic angle, and in turn regulate gene transcription [17]. Sex-determining region Y-box 2 (*Sox2*) is an important member of *Sox* family, which is highly similar in its DNA-binding activity to the *Sry*. Strikingly, the main functions of *Sox2* have been reported predominantly within areas of stem cell biology regulation, cellular reprogramming, and disease initiation and maintenance, especially cancer, but not in sex determination [18]. Recently, *Sox2* was reported to be a target gene of miR-126, and the interaction between miR-126 and *Sox2* was shown to play a key role in gastric carcinogenesis [19]. However the role of miR-126/Sox2 interaction has not been identified in osteosarcoma. Since the involvement of miR-126 in osteosarcoma carcinogenesis is largely unexplored, we have investigated osteosarcoma cell lines under-expressing miR-126, with the aim to study its effects on cellular progressions and to identify the mechanisms involved. In this paper, we explored the expression of miR-126 in 32 formalin-fixed, paraffin-embedded tumor tissues using TaqMan RT-PCR analysis. Subsequently, we completed a series of cellular function experiments to investigate the role of miR-126 in osteosarcoma.

## 2. Results

### 2.1. miR-126 Was under-Expressed in OS Tissues and OS Cell Lines

To explore the expression and significance of miR-126 in OS carcinogenesis, firstly, we detected the expression of miR-126 in 32 pairs of OS tissues and the matched normal tissues by TaqMan RT-PCR analysis. Relative to matched normal tissues, more than half of the OS tissues exhibited under-expression of miR-126 (68.7%, 22 of 32, Figure 1A). Moreover, statistical analysis further identified the under-expression of miR-126 in OS tissues compared with normal tissues (Figure 1B). Furthermore, to identify whether this under-expression only exists in OS tissues, we explored the expression of miR-126 in four OS cell lines (HOS, Saos-2, U2OS and MG-63). Compared with the normal human osteoblast cell line (NHOst), the expression of miR-126 in four OS cell lines was reduced (Figure 1C). These results suggested that the under-expression of miR-126 is a frequent event in human OS.

RETRACTED

### 2.2. miR-126 Functions as a Tumor Suppressor in MG-63 Cells

The under-expression of miR-126 in both human OS tissues and OS cell lines prompted us to explore ist possible biological role in OS carcinogenesis. As miR-126 significantly decreases in OS tissues, we sought to compensate for its loss through exogenous transfection with the miR-126 mimic into MG-63 cells, and the scramble mimic was used as negative control. The intracellular level of miR-126 was about 500-fold higher in MG-63 cells transfected with the miR-126 mimic relative to the scramble control group (Figure 2A). Cell proliferation was then measured using CCK-8 assays. Ectopic expression of miR-126 led to a significant decrease in cell proliferation of MG-63 cells (Figure 2B). As proliferation directly links to cell cycle distribution, the effect of miR-126 on cell cycle progression was analyzed. As expected, the percentage of S phase cells was reduced in MG-63 cells upon transfection with the miR-126 mimic (Figure 1C). Thus, restored miR-126 expression could arrest cell cycle progression and then inhibit cell proliferation.

Given that migration and invasion promote tumor metastasis, which composes the major cause of cancer death, we performed more assays to investigate the effects of miR-126 on cell migration and invasion of MG-63 cells. As shown in Figure 2D,E, restored expression of miR-126 in MG-63 cells resulted in a significant reduction of cells passed through the chambers, suggesting a suppressive effect of miR-126 on cell migration and invasion of MG-63 cells. All cells in these experiments were maintained in serum-free medium to avoid any augmented migratory or invasive behavior affected by altered cell proliferation. Taken together, these results indicated that miR-126 can efficiently inhibit cell progression of MG-63 cells, and function as a tumor suppressor in OS cells.

### 2.3. miR-126 Targets Sox2 in MG-63 Cells

miRNAs regulate the expression of mRNAs by targeting the 3′UTR of relative mRNAs. To explore the mechanisms involved in miR-126-mediated tumor suppression, putative targets of miR-126 were searched using the prediction program, MicroCosm Targets. Among common predicted targets of miR-126, *Sox2* was selected out for its constitutive over-expression in OS. Although a previous work reported that miR-126 inhibited cell growth by targeting Sox2 in gastric cancer, the role of miR-126/Sox2 interaction is less known in OS. As shown in Figure 3A, there exists two putative binding sites of miR-126 in the 3′UTR of *Sox2* gene (102–108 bp, 367–372 bp). To determine whether or not the two putative binding sites perform a function, we performed luciferase assays. The putative 3′UTR of *Sox2* gene was amplified and cloned into a luciferase reporter vector, and the constructs with each binding sites mutated, MUT-1 and MUT-2, or both sites mutated, MUT-12 were used as controls. These constructs were transiently transfected into MG-63 cells, and the transcription activities were measured using a dual-luciferase detection system. As expected, significant repression of luciferase activities were observed in MG-63 cells co-transfected with pGL3-Sox2 3′-UTR vector and miR-126 mimic compared to mutant constructs groups. Each single mutant construct, MUT-1 and MUT-2, exhibited a lower inhibitory effect on luciferase activity compared with the pGL3-Sox2 3′-UTR vector after miR-126 co-transfection, and the double mutant construct, MUT-12, showed complete reversal of inhibitory effect of miR-126 co-transfection (Figure 3B), suggesting that miR-126 suppressed the transcription activity of the *Sox2* gene by targeting the two binding sites in the 3′UTR of Sox2 mRNA independently.

RETRACTED

To further validate the results of prediction, we examined whether or not miR-126 could influence the expression of endogenous Sox2 mRNA and protein. Consistent with the reporter results, we observed that upon transfection with miR-126, the expression of Sox2 protein and mRNA were both decreased relative to the scramble group (Figure 3C,D). Collectively, these findings suggest that miR-126 regulates the expression of *Sox2* post-transcriptionally.

### 2.4. miR-126 Suppresses Cell Progression by Targeting *Sox2*

A previous work has reported the oncogene role of *Sox2* in OS. They found that Sox2 is up-regulated in human and mouse OS cell lines, and suppression of Sox2 through shRNA could drastically reduce the ability to form colonies, migration and invasion *in vitro*, and inhibited tumor growth *in vivo* [15]. Although the target role of Sox2 has been identified, the function of miR-126/Sox2 interaction mediated in OS remains unclear. To explore whether miR-126-mediated growth inhibition in MG-63 cells via direct targeting *Sox2*, we adopted a “rescue” methodology. We generated a new construct containing the full ORF of *Sox2* gene (pcDNA-Sox2). As expected, the level of *Sox2* was rescued when pcDNA-Sox2 was transfected into MG-63 cells that had been treated with miR-126 mimic for 24 h (Figure 4A). In agreement with the restored expression of *Sox2*, increased cell proliferation (Figure 4B), accompanied with decreased cell apoptosis (Figure 4C) were also observed in MG-63 cells transfected with pcDNA-*Sox2* constructs following the treatment of miR-126. Moreover, upon transfection with the *Sox2* construct, the suppression of miR-126-mediated cell migration (Figure 4D) and invasion (Figure 4E) in MG-63 cells was also abolished. Taken together, these results demonstrate that the repression of cell progression by miR-126 was typically a consequence of decreased *Sox2* expression in OS cells.

RETRACTED

## 3. Discussion

The recently discovered miRNA gene regulators represent approximately 1% of the genome of different species [20]. Accumulating evidence has demonstrated the aberrant expression of miRNAs in cancer is not just a random event, but exerts an important role in the tumorigenic processes. Therefore, better understanding of the physiological and disease-associated mechanisms of these small, single-stranded RNAs may provide a new way for diagnosis and therapy of future diseases. In this study, we provide important evidence in support of miR-126 functioning as a tumor suppressor in OS.

Although previous work has reported the under-expression of miR-126 in OS [10], the function and relevant mechanisms of miR-126 in OS have not been identified. To further understand the role of miR-126 in OS, we detected the expression of miR-126 in 32 paired OS tissues and normal bone tissues. As expected, our study validated the under-expression of miR-126 in OS tissues. Moreover, our experiment is consistent with the results of Xu *et al*., which identified the under-expression of miR-126 in four OS cell lines, and that over-expression of miR-126 could inhibit cell proliferation by targeting Sirt1 [21]. These data consistently suggested the tumor suppressor role of miR-126 in OS.

To further validate the tumor suppressor role of miR-126 in OS, we next examined the function of miR-126 on OS cells. As miR-126 significantly decreases in OS tissues and cell lines, we sought to compensate for its loss through exogenous transfection with miR-126 mimic into MG-63 cells. The results shown here demonstrate that miR-126 could suppress the tumorigenicity of OS cells. Restored expression of miR-126 markedly inhibited cell proliferation and induced cell apoptosis. Moreover, miR-126-transfected cells showed a dramatic decrease in cell migration and invasion, accompanied with suppressed expression of *Sox2*, which contains two putative binding sites of miR-126 in its 3′UTR identified by the prediction program MicroCosm Targets. Further, luciferase assays confirmed the function of these two sites; through transfection with miR-126, the expression of Sox2 mRNA and protein were both suppressed. Although Sox2 has been demonstrated to be the target gene of miR-126 in gastric cancer [19], this is the first time to validate the function of miR-126/Sox2 interaction in the progression of OS.

RETRACTED

*Sox2* belongs to the Sex-determining region Y-related high-mobility group box gene family and is a critical transcription factor in embryonic and cancer stem cells [22]. It plays an important role in cell self-renewal, differentiation, proliferation and apoptosis [23,24]. There is accumulating evidence that *Sox2* is overexpressed in various human tumors, such as human lung squamous cell carcinoma, rectal cancer, prostate cancer and so on [25–27]. Moreover, constitutive activation of *Sox2* has been reported to be closely associated with poor survival and metastasis of hepatocellular carcinoma (HCC) patients. By activating Slug transcription activity, *Sox2* induces HCC cell migration and invasion [28]. On the other hand, suppression of Sox2 inhibits cell proliferation and induces cell apoptosis of androgen-independent human prostate cancer cell by targeting cyclinE, p27 and survivin genes, respectively [29]. For OS, *Sox2* has been reported to be highly expressed in human and mouse OS cell lines as well as clinical samples, and suppression of *Sox2* through shRNA-impaired cell growth in soft agar, decreased migration and invasion, and reduced the transformed phenotype of OS cells *in vitro* [30], that means *Sox2* promotes tumorigenesis in OS. Furthermore, genomic analysis of OS, interestingly revealed no activating mutations have been found in the genes encoding the *Sox2* gene [30]. We therefore speculate that the over-expression of *Sox2* in OS might come from an epigenetic dysregulation, rather than an abnormal gene mutation. miRNA mediated-post-transcriptional gene regulation is emerging as an important epigenetic regulation mechanism [6]. In this paper, we found that the activation of *Sox2* might be a consequence of constitutive suppression of miR-126. Moreover, *Sox2* was reported to be the target of miR-29b [31], miR-378 [32], miR-429 [33] and miR-140 [34] recently. Through suppressing the expression of Sox2, these miRNAs mediated important functions in cellular reprogramming, self-renewal, apoptosis and proliferation, respectively, meaning that miRNAs-mediated Sox2 dysregulation might play a critical role in various cellular processes.

Lastly, we restored the expression of Sox2 in miR-126-transfected cells to explore the role of *Sox2* in miR-126-mediated tumor suppression. As expected, restoring the expression of *Sox2* in OS cells, abolished miR-126-mediated suppression, which suggest that *Sox2* might have a key role in miR-126 mediated tumor suppression of OS cells. Taken together, down-regulation of miR-126 in OS cells may contribute to the increasing expression of *Sox2* at the post-transcriptional level and in turn facilitate OS carcinogenesis.

RETRACTED

## 4. Materials and Methods

### 4.1. Patients and Tissue Specimens

32 formalin fixed paraffin-embedded specimens of osteosarcoma tissues were collected from dthe Department of Orthopedic Surgery, the First Affiliated Hospital of Harbin Medical University. The matched normal tissues were obtained 5 cm distant from the tumor margin, which were further confirmed by pathologists. All patients did not undergo any therapy before recruitment to this research. Use of the tissue samples for all experiments was approved by Ethics Committee of the instruction.

### 4.2. Cell Lines and Cell Culture

Human osteosarcoma cell lines (HOS, Saos-2, U2OS and MG-63) or normal osteoblast cells (NHOst) were obtained from the American Type Culture Collection (ATCC, Manassas, VA, USA). The cells were maintained in Dulbecco’s modified Eagle medium (DMEM, Gibco, Life Technologies, Darmstadt, Germany), supplemented with 10% fetal bovine serum (FBS; PAA, Pasching, Austria) and streptomycin (100 μg/mL), penicillin (100 U/mL). Cultures were incubated in a humidified atmosphere of 5% CO_2_ at 37 °C.

### 4.3. RNA Extraction, Reverse Transcription and Quantitative Real-Time PCR

According to the protocol of Recover All Total Nucleic Acid Isolation Kit (Ambion, Austin, TX, USA), total RNA was isolated from 20-μm sections from formalin-fixed, paraffin-embedded tissue blocks. To quantitate the miRNA expression, the expression of small nuclear U6 was used as internal control. Total RNA was reversely transcribed using First-Strand cDNA Synthesis kit (Invitrogen, Carlsbad, CA, USA). Specific primers qualified with a Taqman probe for reverse transcription were used as follows: miR-126: 5′-GTCGTAT CCAGTGCAGGGTCCGAGGTATTCGCACTGGCGCUTT-3′; and U6: 5′-AAAATATGGA ACGCTTCACGAATTTG-3′. Then, quantitative real-time PCR was performed to quantify relative expression of miR-126 using the Quanti-TectSYBR Green PCR mixture on an ABI PRISM 7900 Sequence Detection System (Applied Biosystems, Carlsbad, CA, USA). The primers for qRT-PCR reaction were used as follows: miR-126: sense: 5′-GCUCGUACCGUGAGUA AU-3′; anti-sense: 5′-CAGTGCAGGGTCCGAGGT-3′; U6: sense: 5′-CTCGCTTCGGCAGCACA TATACT-3′; anti-sense: 5′-ACGCTTCACGAATT TGCGTGTC-3′.

For analysis of mRNA expression, total RNA was extracted from cells using the TRIzol reagent (Invitrogen, Carlsbad, CA, USA) according to the manufacturer’s instructions. The expression of GAPDH was used as internal control and Oligo(dT) was used as the primer for Sox2 and GAPDH reverse transcription. Then, quantitative real-time PCR was performed to quantify relative expression of Sox2 with the following primers: Sox2: sense: 5′-GCTACAAGACAACACCCTGAT-3′; anti-sense: 5′-CAATCTCCTAAGCCACGAG-3′; GAPDH: sense: 5′-TCAACGACCACTTTGTCAAGCTCA-3′; anti-sense: 5′-GCTGGTG GTCCAGGGGTCTTACT-3′. PCR efficiencies were calculated with a relative standard curve derived from a complementary DNA mixture and gave regression coefficients >0.95. The relative expression levels were evaluated using the 2^−ΔΔ^*^C^*^t^ method. All experiments repeated three times.

RETRACTED

### 4.4. Cell Transfection

miR-126 mimic and scramble mimic were all purchased from Dharmacon (Austin, TX, USA). All oligonucleotides were transfected into MG-63 cells to a final concentration of 50 nM by Dhamafect 1 (Dharmacon, Lafayette, CO, USA) according to manufacturer’s instructions. Cells were collected for further experiments 48 h post-transfection with miR-126 mimic.

### 4.5. Cell Proliferation Assay

Before analysis of cell proliferation, MG-63 cells were seeded into 24-well plates at a concentration of 5 × 10^3^ cells/well. The Cell Counting Kit-8 (CCK-8, Dojindo, Kumamoto, Japan) was added to the wells at 0, 24, 48, and 72 h post-transfection, and cells were diluted in normal culture medium at 37 °C until visual color conversion occurred. The absorbance values in each well were measured with a microplate reader set at 450 and 630 nM. All experiments were performed three times and the average percentages of cells are shown.

### 4.6. Cell Apoptosis Analysis

For analysis of apoptosis, MG-63 cells were collected and diluted to a concentration of 1 × 10^6^ cells/mL and washed three times with ice-cold PBS 72 h after transfection. Cells were incubated with Annexin V-PE and 7AAD, according to the Annexin V-PE Apoptosis Detection Kit I (BD Pharmingen, CA, USA) protocol, and then analyzed by FACS. Cells undergoing early apoptosis binding only to Annexin V, and cells binding both are either in the late stages of apoptosis or already dead. The experiment was repeated three times.

### 4.7. Cell Migration and Invasion Assays

Migration assays were carried out in modified Boyden chambers (BD Biosciences, San Jose, CA, USA) with 8 μm pore filter inserts in 24-well plates. Twenty-four hours after transfection, 2 × 10^5^ cells suspended in serum-free DMEM were added to the upper chamber. For invasion assays, the transwell migration chambers were coated with Matrigel (BD Biosciences, San Jose, CA, USA) and incubated at 37 °C for 3 h, allowing it to solidify. After 24 h of transfection, 4 × 10^5^ cells suspended in serum-free DMEM were added to the upper chamber. DMEM containing 20% FBS were added to the lower chambers as a chemoattractant. After 24 h transfection, the non-filtered cells were gently removed with a cotton swab. Filtered cells located on the lower side of the chamber were stained with crystal violet, air-dried and photographed. Three independent experiments were performed.

RETRACTED

### 4.8. Plasmid Construction

The full length *Sox2* gene open reading frame (ORF) were amplified by PCR reaction and cloned into pCDNA3.1 construct to generate the pCDNA3.1-Sox2 construct, and the empty pCDNA3.1 construct was used as control. Sequences of primers used for PCR amplification are sense: 5′-AAACGAGGGAAATGGGAG-3′; anti-sense: 5′-TACCAACGGTGTCAACCTG-3′, respectively. MG-63 cells were first transfected with miR-126 mimics or scramble mimics (60 nM) in six-well plates. After 24 h of culture, these MG-63 cells were then co-transfected with miR-126 mimics (30 nM) and 2.0 μg of either pcDNA-Sox2 or pcDNA-3.1. The cells were harvested at predetermined intervals and assayed as necessary.

### 4.9. Luciferase Assays

The whole 3′-UTR of *Sox2* gene was cloned into the pGL-3-vector (Promega, WI, USA) immediately downstream of the *Renilla* luciferase gene. Mutations in the 3′-UTR of *Sox2* gene with miR-126 target sites deleted (Mut A, Mut B or Mut AB) were generated with the QuickChange Site-Directed Mutagenesis kit (Stratagene, CA, USA). About 1 × 10^5^ MG-63 cells per well were seeded into 24-well plates for 24 h before transfection. Cells were co-transfected with 50 ng pGL-3 firefly luciferase reporter, 10 ng pRL-TK Renilla luciferase reporter and 50 nM miR-126 mimics or scramble mimics using Lipofectamine 2000 (Invitrogen, Carlsbad, CA, USA). A luciferase reporter construct containing the miR-126 consensus target sequence served as the positive control and the pRL-TK vector served as the internal control. Cell lysates were prepared using Passive Lysis Buffer (Promega, Madison, WI, USA) 48 h after transfection, and luciferase activity was measured using the Dual-Luciferase Reporter Assay (Promega, Madison, WI, USA). Results were normalized to the Renilla luciferase. Experiments were independently repeated three times.

### 4.10. Western Blot Analysis

For the western blot assay, cells were harvested in ice-cold PBS 48 h after transfection and lysed on ice in cold modified radioimmunoprecipitation buffer supplemented with protease inhibitors. Protein concentration was determined by the BCA Protein Assay Kit (Bio-Rad, Hercules, CA, USA) and equal amounts of protein were analyzed by SDS-PAGE. Gels were electroblotted onto nitrocellulose membranes (Millipore, Billerica, WI, USA). After blocked with 5% non-fat dry milk in Tris-buffered saline containing 0.1% Tween-20 2 h, membranes were incubated at 4 °C over night with primary antibody (Sox2 and GAPDH, Cell Signaling, MA, USA). Then, membranes were incubated with respective second antibodies and detected by peroxidase-conjugated secondary antibodies using the enhanced chemiluminescence system (ECL) (Millipore, Billerica, WI, USA). The experiment was repeated three times.

RETRACTED

### 4.11. Statistical Analysis

Data were expressed as the mean ± standard deviation of at least three independent experiments. Statistical analysis was carried out using SPSS 15.0 software (SPSS Inc.; Chicago, IL, USA). Student’s *t*-test (two-tailed) was performed to analyze the data. *p*-values < 0.05 were considered significant.

## 5. Conclusions

In conclusion, our findings demonstrate that miR-126 acts as a tumor suppressor in OS through targeting *Sox2*. Re-introduction of miR-126 in MG-63 cells can down-regulate *Sox2*, which dampens cell growth, inhibits cell migration and invasion, and induces cell apoptosis, however, all these activities could be suppressed through over-expression of *Sox2*. Collectively, this finding not only furthers our understanding of the molecular mechanisms of OS carcinogenesis, but also provides a strong rationale to further investigate miR-126 as a potential biomarker and therapeutic target for OS.

## Figures and Tables

**Figure 1.** The expression of miR-126 in osteosarcoma tissues and cell lines. (**A**) The expression of miR-126 in 32 pairs of OS tissues and adjacent normal bone tissues was detected by TaqMan quantitative RT-PCR. Data are shown as log10 of relative ratio change of OS tissues relative to normal bone tissues. 68.7% of the patients showed the under-expression of miR-126 relative to normal tissues; (**B**) Statistical analysis of relative miR-126 expression levels in OS tissues and compared normal tissues. Compared with normal bone tissues, the expression of miR-126 in tumor tissues was significantly down-regulated; and (**C**) Using RT-PCR analysis, the expression of miR-126 in four OS cell lines (HOS, Saos-2, U2OS and MG-63) was analyzed. The expression of miR-126 in these OS cell lines was under-regulated relative to normal osteoblast cells (NHOst). ** *p <* 0.01; *** *p <* 0.001 compared with normal tissues or normal osteoblast cells.

**Figure 2.** miR-126 suppresses OS tumor progression. (**A**) RT-PCR was performed to detect the expression of miR-126 in OS cell line MG-63 after treatment with mimic. Upon transfection with the miR-126 mimic, the expression of miR-126 in MG-63 cells was restored; (**B**) CCK-8 was performed to analyze the effect of miR-126 on cell proliferation of MG-63 cells. Ectopic expression of miR-126 inhibited cell proliferation; (**C**) The influence of miR-126 on cell apoptosis was analyzed using cell apoptosis assays. Transfection with miR-126 showed more cells undergoing early apoptosis; and (**D**,**E**) The effects of miR-126 on cell migration and invasion were detected using transwell chamber assays. Panel D showed the results on migration. Over-expression of miR-126 dampened cell migratory capacity with suppressing cells passed through the membrane; Panel E showed the results on invasion. The chambers have been coated with Matrigel, which functions as the extracellular cell matrix. miR-126 inhibited cells invasion through the membrane. (×100); * *p <* 0.05; ** *p <* 0.01; *** *p <* 0.001 compared with scramble group.

RETRACTED

**Figure 3.** miR-126 targets the Sox2 gene in MG-63 cells. (**A**) Schematic representation of Sox2 3′UTR showing putative miRNA target sites. There exist two putative binding sites in the 3′UTR of miR-126; (**B**) Relative luciferase activity of the indicated Sox2 reporter construct in MG-63 cells, co-transfected with miR-126 mimics or scramble mimics, is shown. In cells co-transfected with pGL3-Sox2 3′-UTR vector and miR-126 mimic, the luciferase activity was suppressed relative to mutant construct groups, and the one in both binding sites mutant (MUT-12) showed the lowest activity; and (**C**,**D**) Quantitative RT-PCR and Western blot assays were performed to detect the expression of Sox2 upon transfection with miR-126 mimics or scramble mimics. The expressions of mRNA and protein were suppressed upon transfection with miR-126. ** *p <* 0.01 compared with scramble group.

**Figure 4.** miR-126 suppresses tumor progression through targeting Sox2. (**A**) Upon transfection with Sox2 construct, we rescued the expression of Sox2 in MG-63 cells. The expression of Sox2 protein was validated by western blot assays; (**B**) CCK-8 assays were used to detect in MG-63 cells co-transfected with miR-126 mimic and pcDNA-Sox2 plasmid; (**C**) Cell apoptosis of MG-63 cells treated as described in B was detected by Annexin V-PE staining; and (**D**,**E**) Transwell assays were performed to detect the effects on cell migration and invasion of MG-63 cells treated as described in B. Upon transfection with the Sox2 plasmid, miR-126-mediated suppression of cell proliferation, cell migration and invasion was abolished, and promotion of cell apoptosis was inhibited. (×100); * *p <* 0.05 compared between two groups as shown with a line.
